# Analysis of the Effect of Emergency Ventilators on the Treatment of Critical Illness Based on Smart Medical Big Data

**DOI:** 10.1155/2021/7698769

**Published:** 2021-09-21

**Authors:** Haiwang Sha, Fen He

**Affiliations:** Department of Critical Care Medicine, Yanan University Affiliated Hospital, Shaanxi 716000, China

## Abstract

Respiratory failure refers to pulmonary ventilation and ventilatory dysfunction caused by various reasons, which makes the patient unable to maintain the gas exchange required for stillness and causes a series of pathophysiological changes and corresponding clinical manifestations. In order to solve the problem of respiratory failure in critically ill patients, it is of great significance to analyze the role of microprocessor-based emergency ventilator in the treatment of critically ill patients. This article aims to study the role of microprocessor-based emergency ventilator in the treatment of critically ill patients. This paper presents the key technology based on the ARM11 processor. A breathing motion model is detected and established through a ventilator. The research objects are mainly divided into group A and group B. By comparing the two groups of emergency ventilator ventilation, it can effectively prevent the increase in respiratory muscle fatigue, reduce oxygen consumption, improve the patient's ventilation function and oxygen balance, quickly correct hypoxia and carbon dioxide storage, cooperate with drug treatment, and quickly take out the ventilator after relief. Good treatment results were achieved. The results show that the emergency ventilator controlled by a microcomputer is effective. The total effective rate of the control group was 71.11%, which was significantly lower than that of the observation group (86.67%).

## 1. Introduction

### 1.1. Background

Respiratory failure refers to pulmonary ventilation and/or ventilatory dysfunction caused by various reasons, so that the patient cannot maintain the gas exchange required during rest, resulting in hypoxemia with (or without) hypercapnia and then causing a series of pathophysiological changes and corresponding clinical manifestations. Domestic research mainly focuses on the detection of virus types in outpatients and ordinary inpatients, or the detection of patient-specific virus antibodies. There are few viral etiology analyses in patients with respiratory failure in ICU in China. One hundred and sixteen pathogenic bacteria isolated from ICU patients in large hospitals in China were analyzed. Gram-negative bacilli accounted for 57.8%, fungi accounted for 30.2%, and Gram-positive cocci accounted for 12.1%. These studies only analyzed the pathogen distribution of bacteria and fungi but did not detect and analyze the pathogens of viruses.

### 1.2. Significance

Respiratory failure is one of the most common causes of death in ICU. The risk of death in the intensive care unit is higher, and it is also a common disease in the ICU. Infectious factors are the most common cause of pulmonary respiratory failure. Ventilator is necessary rescue equipment in large hospitals, and it is an important means to prolong the lives of patients and gain valuable time for further treatment. With the continuous progress of electronic mechanical technology, the performance of the ventilator is improving day by day, and its application scope is also expanding and popularizing. This study aims to explore the role of computerized emergency ventilator in the treatment of acute and severe diseases.

### 1.3. Related Work

The ventilator is necessary rescue equipment in large hospitals. It is an important tool to prolong the lives of patients and gain valuable time for further treatment. Schiffl H pointed out that acute kidney injury is a heterogeneous clinical syndrome, including a variety of risk factors and acute injury, which occurs in a variety of situations and will affect short-term and long-term results. Obesity has become an epidemic. The existing literature shows that AKI is very common in patients with severe surgery or medical obesity, and obesity is a new risk factor for this acute renal syndrome. The pathophysiology of obesity-related AKI is not fully understood. Obesity-related factors plus the burden of other comorbidities in elderly obese patients may interact with known precipitating factors (such as hypotension, nephrotoxin, or sepsis) and increase the population's susceptibility to AKI. Whether obesity may be protective against intuition and is associated with better survival of patients with severe AKI (reverse epidemiology) is a controversial topic. There is an urgent need to further study the role of new biomarkers and the best management, but more research is needed to further find the best management method [1]. Ren pointed out that the downgrade strategy is to gradually transition various complex, expensive, high-risk, but effective treatments for severely ill patients to simple, safe, physiological, but still effective treatments. Chronic critical illness refers to a patient who is in a serious condition or is hit by an operation, turns into a chronic relapse or even aggravated state, and stays in the intensive care unit for a long time. Risk factors for chronic critical illnesses associated with surgery include advanced age, malnutrition, multiple organ dysfunction, and multiple blows. In the treatment of critically ill patients, degrading treatment strategies should always be implemented, including rational use of antibiotics, degrading fluid therapy (i.e., deresuscitation), timely removal of the ventilator, rapid introduction and withdrawal of the ventilator, continuous renal replacement measures, parenteral + enteral nutrition support treatment, and stopping sedation in time. However, he did not comment on the timing of stopping sedation [2]. Zhu pointed out that, with the development of society and economy, people's requirements for emergency rescue technology and emergency services have gradually increased. Establishing and improving the emergency situation of the intensive care system is an important issue currently faced. Controlling medical injuries is the goal of medical development. At present, people's requirements for first aid measures have shown a trend from invasive to minimally invasive and even noninvasive. The establishment of a minimally invasive emergency system and the application of minimally invasive technology in the field of emergency and intensive care are the new requirements of emergency medicine in the new era, but it is currently lacking [3].

### 1.4. Main Content

This paper mainly studies the classification processing of emergency ventilator based on microprocessor. This article introduces the advanced features and key technologies of ARM11 processor [4] in emergency ventilator. A polynomial breathing motion model was used to analyze the breathing motion process of the individual after the primary disease caused respiratory failure, and the emergency treatment methods were analyzed. Through research experiments, the research objects are investigated and analyzed, so that patients and their families can understand the safety and feasibility of the research, do a good job in patients' ideological work, reduce the psychological burden of patients, and gain the understanding and cooperation of patients and their families. A consent form for voluntary participation in this clinical trial was obtained. In the experiment, the basic conditions of patients before and after grouping were compared and analyzed, and the effect of phased treatment based on the microprocessor-based emergency ventilator was summarized.

## 2. Key Technologies and Methods

### 2.1. Features and Key Technologies of Arm11 Processor

#### 2.1.1. Key Technologies and Core Features

The ARM11 series microprocessor is the next-generation RISC processor developed by Arm Company in recent years [5, 6], which is the design and application of the first generation Armv6. The new ordered architecture includes three models of arma1136i, arma1156t2, and arma1176jz. The first step is to improve the understanding of next-generation microprocessors for different application fields and establish a new architecture. The processor does not specify the configuration of the processor. The system structure is defined to provide an interface between the processor and the outside. Environment (operating system, application support, and debugging) programming method and final memory.

#### 2.1.2. Excellent Performance of ARMv6 Processor

In general, the ARMv6 architecture enhances the performance of the processor through the following points:

1. Multimedia processing extension. It doubles the speed of MPEG4 encoding/decoding and the speed of audioprocessing.
2. Enhanced cache structure. real address cache, reduces the cache refresh and reload, and reduces the overhead of context switching.
3. Enhanced exception and interrupt handling. It makes real-time task processing faster, supports unaligned and mixed-end data access, makes data sharing and software migration easier, and helps save memory space. For most applications, ARMv6 maintains 100% binary downward compatibility, so users can further inherit programs developed in the past. Armv6 retains all the extensions of T (thumb instruction [7]) and E (DSP instruction) in the previous architecture, thus continuing the characteristics of code compression and DSP processing; in order to speed up the execution of Java code, ARM Jazelle technology continues to be used in the ARMv6 system and plays an important role in the structure.

### 2.2. Detecting and Establishing the Type of the Breathing Motion Model

#### 2.2.1. Piecewise Linear Breathing Motion Model

In this case, the tissue movement is represented by multiple images, and each image corresponds to a different substitute signal value. These motion parameters are linearly interpolated to estimate the motion at the alternative signal that has not yet been acquired. Such a model allows tissue movement to follow more complex trajectories instead of simple straight lines. However, with a single substitute signal, the simulation error of these models will be limited. A piecewise linear respiratory motion model that correlates motion with measured substitute signals cannot simulate respiratory lag but can simulate some errors between respiratory cycles.

#### 2.2.2. Tissue Breathing

The time always follows the same movement trajectory, but the distance of movement under this trajectory can be different, depending on the depth of breathing of the patient. The piecewise linear respiratory motion model that correlates motion and respiratory phase can simulate respiratory lag but cannot simulate the error between respiratory cycles. In addition, it is not possible to construct a piecewise linear respiratory motion model with a substitute signal value beyond the measurement range [8].

The polynomial breathing motion model constructed by using a single scalar to replace the signal s1 is as follows:

(1) $$\begin{array}{c} M=\sum_{i=0}^{q}C_{i}s_{1}^{i}. \end{array}$$

The polynomial respiratory motion model constructed by using two scalar substitute signals s1 and s2 is as follows:

(2) $$\begin{array}{c} M=\sum_{i=0}^{q}\sum_{j=0}^{n-i}C_{i,j}{\text{s}}_{1}^{i}s_{2}^{j}. \end{array}$$

Among them, *C*_*i*,*j*_ and are polynomial coefficient vectors, and *q* is the polynomial order. The motion model is usually a second-order or third-order polynomial breathing motion model. Higher-order polynomials have also been studied, but higher-order polynomials are more prone to overfitting, leading to large extrapolation errors.

Polynomial respiratory motion models usually only use a single scalar to replace the signal, but some also use respiratory phase at the same time, just like a linear respiratory motion model. If only one substitute signal is used, although the length of the motion trajectory will be different, it still follows the same motion trajectory. Unlike the linear breathing motion model, the motion trajectory is no longer a straight line. Since the polynomial breathing motion model can easily lead to large extrapolation errors, when estimating the motion at the substitute signal value outside the measurement range, some studies reselect the linear equation to construct the motion model.

The polynomial breathing motion model constructed with a single substitute signal cannot simulate hysteresis, because it is restricted to move on the same trajectory during inhalation and exhalation.

#### 2.2.3. B-Spline Breathing Motion Model

The respiratory phase extracted from a single signal is used as a substitute signal to construct a one-dimensional B-spline respiratory motion model. There are also studies using actual measurement signals and extracted respiratory phase signals to construct a two-dimensional B-spline respiratory motion model. Because of the correlation between internal tissue movement and respiratory phase, most articles have modified the standard B-spline function [9] to make it a periodic function, which can eliminate discontinuities between respiratory cycles.

(3) $$\begin{array}{c} M=\sum_{i=0}^{3}C_{i+k\mathrm{mod}N}B_{i}\left(j\right). \end{array}$$

Among them *j*=*α*/*β* − [*α*/*β*], *K*=[*α*/*β*] − 1, *α* is the respiratory phase (between 0 and 100%), and *B*_*i*_ is the *i*-th B-spline basis function:

*B*_0_(*t*)=(−*t*^3^+3*t*^2^ − 3*t*+1)/6, *B*_1_(*t*)=(3*t*^3^ − 6*t*^2^+4)/6, *B*_2_(*t*)=(−3*t*^3^+3*t*^2^+3*t*+1)/6, *B*_3_(*t*)=*t*^3^/6, where 0 ≤ *t* ≤ 1. C0 and CN (containing *N* elements) are B-spline control point vectors, and *N* is the number of control points. *α*(*α*=100%/*N*) are the control point spacing. It is worth noting that although the equation is directly related to the motion and the measured replacement signal, the value of the B-spline basis function *B*_*i*_ still depends on the value of the respiratory phase extracted from the measured signal *α*.

The one-dimensional periodic B-spline breathing motion model makes the anatomical structure motion follow the circular trajectory [10], which also means that it can simulate hysteresis but cannot simulate the error between cycles. The two-dimensional B-spline respiratory motion model can simulate the error and hysteresis between cycles, but because there are more model parameters that need to be fitted, there is a risk of data overfitting.

### 2.3. Fitting Method of the Breathing Motion Model

Several different methods and techniques have been used to fit clinical data to obtain respiratory motion models of human internal organs and tissues. This section will introduce some commonly used methods.

In order to fit the respiratory motion model, the motion of the internal anatomical structure at some time points and the replacement signal must be collected at the same time, and each sample point represents a specific time point. At each time sample point *t*, the motion of the internal anatomical structure is represented by the motion vector *M*_*t*_=[*M*_1,*t*_, *M*_2,*t*_,…,*M*_*N*,*t*_]^*T*^, and there are *N* values representing the internal motion (for example, if the motion is represented by the deformation field, then, *N* is three times the number of voxels). At the sample time point *t*, the substitute signal is represented by another vector *S*_*t*_=[*S*_1,*t*_, *S*_2,*t*_,…,*S*_*N*,*t*_]^*T*^, in which there are *N* substitute signals. All motion data samples can be connected to form a matrix *m*=[*M*_1_, *M*_2_,…, *M*_*N*_], and all substitute signal samples can be connected to form another matrix *s*=[*s*_1_, *s*_2_,…, *s*_*N*_], where N is the number of training samples, that is, the number of internal motion time points collected. If 4D lung CT images are used to show internal movement, it is usually 8 or 10, and if different scanning modes are used [11], *N* will be more.

#### 2.3.1. Linear Least Squares Method

So far, the most commonly used method is the linear least squares method [12]. The breathing motion model can be transformed into a linear multiple regression problem:

(4) $$\begin{array}{c} M_{t}=Cs_{t}. \end{array}$$

*C* contains the respiratory motion model parameters. These parameters can be calculated from the training data by using ordinary least squares to minimize the squared difference between *M* and *Cs*, namely,

(5) $$\begin{array}{c} \arg\;\min{\left(m-Cs\right)}^{2}. \end{array}$$

This can be obtained by

(6) $$\begin{array}{c} C=mS^{T}{\left(SS^{T}\right)}^{-1}=\sum_{MS}\sum_{SS}^{-1}. \end{array}$$

Among them, ∑_*SS*_ is the covariance matrix of *S*, and ∑_*MS*_ is the cross-covariance matrix of *M* and *S* [13].

For motion estimation *M*_*est*_, the new replacement signal value *s*_new_ can be used to obtain the parameter *C* of the fitted breathing motion model.

(7) $$\begin{array}{c} M_{est}=Cs_{\text{new}}. \end{array}$$

The linear least squares method is widely used, the principle is simple, and it is easy to implement.

#### 2.3.2. Principal Component Analysis Method

It can be used to help analyze and interpret multivariate data. The number of principal components is the same as the number of variables in the data. However, usually not all the principal components are used, but a smaller number of principal components can retain the original data information at most. Therefore, the principal component analysis method can reduce the dimensionality of the original data. The original data can be reexpressed according to the weight of the principal components. If all principal components are used, it is only an approximation of the original data. Principal component analysis is used in different ways to fit the respiratory motion model [14]. Fit the breathing motion model.

Principal component analysis can also be used to fit respiratory motion models. Combine all the average centered motion vectors and the replacement signal vector to form a single data vector *z*_*t*_=[*m*_*t*_^*T*^, *s*_*t*_^*T*^]^*T*^ of length *N*_*m*_+*N*_*s*_. Then, use the principal component analysis method to act on the matrix *Z* of size (*N*_*m*_+*N*_*s*_) × *N*_*t*_, which contains the data vector extracted from the *N* training samples.

(8) $$\begin{array}{c} Z\approx E_{z}W_{z}, \end{array}$$

where matrix *E*_*z*_ contains the first *K*_*z*_ principal components. The equation can be divided into two independent equations:

(9) $$\begin{array}{c} M\approx E_{zm}W_{z},\\ S\approx E_{zs}W_{z}, \end{array}$$

where *E*_*zm*_ and *E*_*zs*_ are, respectively, composed of the upper *N*_*m*_ rows and the lower *N*_*s*_ rows of *E*_*z*_. Assuming that the inverse matrix *E*_*zx*_^−1^ exists, then, *W*_*z*_ can be obtained from

(10) $$\begin{array}{c} M\approx E_{zs}E_{zs}^{-1}S. \end{array}$$

Remove the estimated motion using the new replacement signal value:

(11) $$\begin{array}{c} m_{est}=m+E_{zm}E_{zs}^{-1}\left(s_{\text{new}}-s\right). \end{array}$$

It should be noted that, for *E*_*zs*_^−1^ to exist, the number of rows in *E*_*zm*_ should be at least equal to the number of columns; that is, the number of principal components used, *K*_*z*_, cannot exceed the number of alternative signals used.

The principal component analysis method [15] can eliminate the relevant influence between data at different times, and the calculation is relatively standardized, which is convenient for computer implementation, but it will lose part of the original information, which is not as clear and accurate as the meaning of the initial data.

## 3. Research Experiment

### 3.1. Research Objects

From December 2020 to May 2021, 48 patients with primary respiratory failure were admitted to the respiratory intensive care unit of our hospital, including 28 males and 20 females. They belonged to the mechanical ventilation group. Of 48, 37 patients had a chronic obstructive pulmonary disease with acute exacerbation of respiratory failure, five patients had a severe pneumonia, six patients had a cerebral hemorrhage or cerebral infarction combined with pulmonary infection and respiratory failure, and all were treated with invasive mechanical ventilation and nasal endotracheal intubation, comprehensive treatment of infection, and nutritional support. The patient's condition is stable, his lung infection is basically controlled, and he can breathe spontaneously. Three spontaneous breathing tests failed. It was difficult to get off the line. Certain respiratory support conditions were still needed.

### 3.2. Test Grouping

The subjects were randomly divided into groups A and B. There was no significant difference in age and gender composition ratio between the two groups (*P* > 0.05). There was no significant difference in arterial blood gas analysis between the two groups (*P* > 0.05):

1. *Group A.* The patient used a noninvasive ventilator before extubation, connected the tracheal intubation extension tube (anesthesia ventilator tubing) through the simple ventilator one-way valve, and connected the tracheal intubation for invasive mechanical ventilation. After the patient adapts, the tracheal intubation is removed, followed by noninvasive mechanical ventilation, and then, the oxygen is inhaled with a nasal cannula.
2. *Group B.* After the patient reaches the condition of weaning, the tracheal intubation is removed. Noninvasive mechanical ventilation is used sequentially [16], and the use time of the noninvasive ventilator is gradually reduced. Then, the nasal cannula is used to inhale oxygen.

### 3.3. Test Procedure

The subjects reached the indicators of group A before weaning. The arterial blood gas analysis was performed two hours before noninvasive mechanical ventilation, and the pH value, PaO_2_, PaCO_2_, and SaO_2_ of the arterial blood gas analysis were recorded.

Choose a well-working noninvasive ventilator (flexo-st30), turn on the noninvasive ventilator, set the parameters of the noninvasive ventilator, select ST mode, and set the positive end-inspiratory pressure of the noninvasive ventilator according to the original parameters of the noninvasive ventilator.

Correctly connect the noninvasive ventilator pipeline, remove the nasal mask or oronasal mask at the end of the noninvasive ventilator pipeline [17], connect the noninvasive ventilator pipeline to the simple respirator one-way valve, and pay attention to the simple respirator one-way valve direction. Disconnect the invasive ventilator pipeline, connect the one-way ventilation valve to the tracheal intubation extension tube (anesthesia ventilator pipeline), and then, connect the tracheal intubation. The noninvasive ventilator and the nasal endotracheal intubation are smoothly connected. The one-way valve of the simple respirator has an oxygen inhalation side hole, which is connected to the central oxygen supply device through an oxygen inhalation tube. The setting of oxygen flow in ECG monitoring is mainly adjusted according to finger pulse oxygen saturation.

During the noninvasive mechanical ventilation with noninvasive ventilator, closely observe the general condition of the patient, including the degree of cooperation between the patient and the noninvasive ventilator, sputum condition [18], changes in finger pulse blood oxygen saturation, and changes in the patient's mood. Do a good job in patient psychological consultation, guide the patient to breathe, and keep the man–machine synchronization. The arterial blood gas analysis was closely monitored, and the arterial blood gas analysis was performed two hours and 24 hours after noninvasive mechanical ventilation.

## 4. Phased Treatment

### 4.1. Basic Situation of the Patients before Grouping

From December 2020 to May 2021, 43 patients were hospitalized in the ICU, including 30 males and 13 females, and 43 patients participated in the entire clinical trial. In the anterior arterial blood gas analysis between the two groups, there were no significant differences in gender, age, degree of disease, pH, PaCO_2_, PaO_2_, and SaO_2_ (see Table 1).

#### 4.1.1. Observing the Changes of Arterial Blood Gas Analysis in Group A Two Hours before and after Noninvasive Mechanical Ventilation

Patients in group A retained the nasal endotracheal intubation and used a noninvasive ventilator instead of an invasive ventilator. Invasive mechanical ventilation was performed. Arterial blood gas analysis was performed two hours before and after treatment. PH and PaO_2_ did not decrease significantly. PaCO_2_ was not significantly retained, and SaO_2_ was maintained well. The difference was not statistically significant (*P* > 0.05) (see Figure 1).

#### 4.1.2. Patients in Group A Kept the Tracheal Intubation, Patients in Group B Removed the Tracheal Intubation, and the Blood Gas Analysis Changed after Using the Noninvasive Ventilator for Two Hours

After reaching the conversion index, group A retained the tracheal intubation and replaced the invasive ventilator with a noninvasive ventilator for invasive mechanical ventilation. In group B, the tracheal tube was removed, and sequential noninvasive mechanical ventilation was used with an oral-nasal mask or a nasal mask. The arterial blood gas analysis was performed two hours after the conversion. The results showed that pH, PaO_2_, PaCO_2_, and SaO_2_ were maintained well, and the difference was not statistically significant (*P* > 0.05) (see Table 2).

#### 4.1.3. The Tracheal Intubation Was Retained in Group A, the Tracheal Intubation Was Removed in Group B, and the Blood Gas Analysis Changed in the Two Groups after 24 Hours of Using the Noninvasive Ventilator

In group A, noninvasive mechanical ventilation was used instead of invasive mechanical ventilation. A 24-hour arterial blood gas analysis showed that pH, PaO_2_, PaCO_2_, and SaO_2_ were maintained well. In group B, a noninvasive ventilator was used after extubation. A 24-hour arterial blood gas analysis showed that the pH value changed, SaO_2_ and PaO_2_ decreased, and PaCO_2_ increased. The difference was statistically significant (*P* < 0.05) (see Table 3).

Changes in relevant indicators of 43 patients with severe asthma before and after mechanical ventilation treatment All patients after mechanical ventilation treatment, the respiratory indicators and blood gas analysis results were significantly improved, as shown in Table 3. Among them, the patient's heart rate, respiratory rate, and partial pressure of carbon dioxide were significantly lowered, and oxygen saturation [19, 20], pH, and partial pressure of oxygen were significantly increased. The differences were statistically significant (0.05). Although the systolic blood pressure has declined compared with the previous one, the difference is not statistically significant. The result is shown in Figure 2.

After extubation, the comparison of the indicators of patients in the sequential noninvasive ventilation group and the nonsequential noninvasive ventilation group also showed that patients were further given sequential noninvasive mechanical ventilation therapy [21], their invasive ventilation and total mechanical ventilation ventilation, hospitalization time, and the incidence of VAP were significantly reduced, and the difference was statistically significant (*P* < 0.05). See Table 4.

CT examination was performed. The control group successfully passed the inspection (22 patients), and the completion rate was 80%. The observation group passed the inspection successfully (25 patients), and the completion rate was 96%. The difference was statistically significant (*P* < 0.05). The observation group's satisfaction (100%) was better than that of the control group (76%), and the difference was statistically significant (*P* < 0.05). See Table 5.

#### 4.1.4. Comparison of Respiratory Support Methods between the Two Groups

The total effective rate of treatment in the control group was 70.11%, which was significantly lower than the 85.67% of the observation group. The difference in the total effective rate of the two groups of patients was statistically significant (*P* < 0.05), as shown in Figure 3.

The proportion of patients in the observation group, who were given resuscitation position, ventilator oxygen, open airway, cricothyrocentesis [22], mask oxygen, nasal cannula oxygen and tracheal intubation, and so on, is not statistically different from the control group [23] (*P* < 0.05), as shown in Table 6.

### 4.2. Distribution of Pathogenic Bacteria and the Status of Specimens Submitted for Inspection

During the two years in our hospital, RICU isolated 559 nonrepetitive strains, of which 364 were derived from sputum (65.1%), 78 strains (14%) from bronchoscopy lavage fluid samples, and 53 strains (9.5%) from blood samples and urine. There were 32 specimens (5.7%): 25 specimens (4.5%) of secretions and seven specimens (1.2%) of pleural effusion and stool. See Figure 4.

The RICU in our hospital collected 559 pathogenic bacteria, 443 Gram-negative bacteria, accounting for 79.2%, 57 Gram-positive bacteria, accounting for 10.2%, and 59 fungi, accounting for 10.5%. The distribution of the main pathogens is shown in Figure 5.

### 4.3. Analysis Results

In recent years, studies have found that adaptive support ventilation and positive end-expiratory pressure ventilation with low tidal volume and low airway pressure can reduce complications and mortality in severe asthma. However, invasive mechanical ventilation combined with some invasive treatment measures can still lead to increased complications, such as hypotension, pneumothorax, emphysema mediastinum [24], atelectasis, arrhythmia, breathing, and related pneumonia (VAP). In most patients, malnutrition and ventilator atrophy lead to prolonged weaning time and difficulty, thereby increasing the risk of death. VAP occurred in two of 43 patients. With the improvement of ventilator function and performance, ventilation method, and nasal mask, noninvasive positive pressure ventilation has shown a good therapeutic effect on respiratory failure caused by various reasons. BiPAP can provide positive pressure assisted ventilation in two ways. After sequential noninvasive mechanical ventilation, the incidence of invasive ventilation, total mechanical ventilation, hospital stay, and VAP [25] were significantly reduced, and the difference was statistically significant (*P* < 0.05). It fully embodies the superiority of the microprocessor-based first aid ventilator, is an effective offline program, and has certain clinical practical value.

## 5. Conclusions

Severe acute asthma includes severe acute-onset asthma, persistent asthma, and refractory asthma. The incidence of asthma has been rising in the past few years. In the acute exacerbation of asthma, although most patients can get some improvement after regular oxygen therapy, systemic application of corticosteroids, powerful bronchodilators, and other drugs, nearly 4% of the patients will continue to get worse. Maintenance therapy with mechanical ventilation is needed to survive the acute phase. Studies have shown that mechanical ventilation can effectively prevent the aggravation of respiratory muscle fatigue, reduce oxygen consumption, improve the patient's ventilation function and oxygen balance, quickly correct hypoxemia and carbon dioxide storage, cooperate with drug treatment, and quickly withdraw after the condition is relieved The ventilator can obtain good therapeutic effects, which is consistent with our research results. The microprocessor-based emergency ventilator has a significant effect. The timely and appropriate implementation of respiratory support for patients with severe asthma is an effective treatment strategy with high rescue success rate and good prognosis.

## Figures and Tables

**Figure 1:** Changes in blood gas analysis of group A before and after the use of noninvasive ventilator with tracheal intubation reserved for two hours.

**Figure 2:** Changes of respiratory index and blood gas analysis of two patients before and after ventilator treatment.

**Figure 3:** Comparison of clinical efficacy and patient satisfaction between the two groups of patients (%).

**Figure 4:** Proportion of nonrepetitive strains and plant tree.

**Figure 5:** Proportion of pathogens.

**Table 1:** General information of the two groups of patients.

	Group A (*n* = 24)	Group B (*n* = 24)	*P*
Gender (female/male)	8/16	10/14	*P* > 0.05
Age	67.10 ± 8.88	67.2 ± 7.73	*P* > 0.05
With tracheal intubation	1	1	*P* > 0.05
History of noninvasive ventilator use	1	2	*P* > 0.05
Adhering to home oxygen therapy	7	6	*P* > 0.05
PH	7.39 ± 0.05	7.40 ± 0.07	*P* > 0.05
PaCO_2_	43.10 ± 3.03	43.3 ± 4.14	*P* > 0.05
PaO_2_	95.40 ± 10.92	95.80 ± 11.45	*P* > 0.05
SpO_2_	94.50 ± 4.25	93.8 ± 4.37	*P* > 0.05

**Table 2:** The changes of blood gas analysis in group A with tracheal intubation retained and group B after extubation using a noninvasive ventilator for two hours.

Group	PH	PaCO_2_ (mmHg)	PaO_2_ (mmHg)	SaO_2_ (%)
Group A	7.39 ± 0.06	43.90 ± 2.92	93.00 ± 5.93	94.20 ± 3.26
Group B	7.38 ± 0.05	43.60 ± 2.07	92.50 ± 5.98	93.80 ± 3.22
*t*	0.73	0.16	0.25	0.60
*P*	>0.05	>0.05	>0.05	>0.05

**Table 3:** Changes in the blood gas analysis after the tracheal intubation retained in group A and the noninvasive ventilator used for extubation in group B for 24 hours.

Group	PH	PaCO_2_ (mmHg)	PaO_2_ (mmHg)	SaO_2_ (%)
Group A	7.40 ± 0.32	43.50 ± 2.27	95.50 ± 3.18	94.8 ± 3.29
Group B	7.35 ± 0.39	49.40 ± 4.45	91.00 ± 1.70	92.66 ± 2.88
*t*	4.00	4.59	3.95	2.80
*P*	>0.05	>0.05	>0.05	>0.05

**Table 4:** Comparison of treatment status of patients in different treatment groups (d).

Parameter	Invasive + noninvasive group (*n* = 22)	Innovative group	*P*
Invasive ventilation time	2.13 ± 0.35	6.25 ± 2.14	<0.05
Total mechanical ventilation time	4.36 ± 1.04	6.05 ± 2.05	<0.05
Hospital stay	9.13 ± 3.24	14.16 ± 4.12	<0.05
VAP	0	2	<0.05

**Table 5:** Satisfaction of the two groups of patients (*n*, %).

Group	*n*	Very satisfied	Satisfaction	Dissatisfied	Total satisfaction
Control group	30	12	10	7	76
Observation group	30	19	11	0	100

**Table 6:** Comparison of respiratory support methods between the two groups (%).

Group	Number of cases	Recovery position	Ventilator oxygen	Open airway	Cricothyrocentesis	Mask oxygen	Nasal cannula oxygen	Tracheal intubation
Observation group	45	15 (33.33)	1 (2.22)	38 (84.44)	16 (35.56)	12 (26.67)	10 (22.22)	2 (4.44)
Control group	45	13 (28.89)	1 (2.22)	39 (88.54)	18 (40.00)	11 (24.44)	9 (20.00)	4 (8.89)
*X*^2^ value		0.199	0.000	3.482	1.916	0.817	0.223	0.266
*P* value		0.351	1.000	0.297	0.099	0.191	0.081	0.267

## Data Availability

Simulated experiment data used to support the results of this research available with periodical reviewers, which can be uploaded.
